The article "Communication Channels for the Rule of Law and Environmental Sustainability: Reflections from a Green Economy Perspective" was published in 2022. Journal: J Environ Public Health.

# Communication Channels for the Rule of Law and Environmental Sustainability: Reflections from a Green Economy Perspective

**DOI:** 10.1155/2022/1811896

**Published:** 2022-09-05

**Authors:** Wen Wen

**Affiliations:** Finance and Economics College, Wanjiang University of Technology, Ma'anshan, Anhui 243031, China

## Abstract

To realize the sustainable development of the environment from the perspective of green economy, it is necessary to effectively utilize the communication channels of environmental sustainability under the rule of law. As a new driving force for economic growth and ecological environment, green economy is analyzed from the perspective of coordinating economic and environmental development. This paper fully analyzes the impact of green economy on economic growth and ecological environment. Based on the inherent relationship, the rule of law and environmental sustainability are conducive to promoting economic growth and also play a continuous role in environmental improvement. Areas with a high level of economic development also have a higher proportion of resource consumption. Driven by technological innovation, green economy can effectively reduce the impact of the environment, promote sustainability, and further promote the coordinated development of the economy and the environment. The results of the case analysis show that, in the proportion of the green economy with a large amount of investment, compared with the traditional policies and regulations, it greatly reduces the aggravation of environmental sustainability and has a positive role in promoting the long-term development of the Chinese economy. It can not only effectively accelerate economic growth, but also realize the reflection from the perspective of green economy and promote the optimization of economic structure.

## 1. Introduction

Real-time, rational, and precise monitoring of ecological environment improvement can also provide a theoretical basis for the decision-making analysis of relevant environmental protection inspection departments, which is of great significance to the continuous emergence of more environmental sustainability improvements. It can be used for detailed analysis of environmental sustainability of ecological environment improvement. In the process of traditional ecological environment improvement evolution analysis, ecological environment improvement and real-time risk alarm are also effective data collection and analysis processes for ecological environment improvement equipment [1, 2]. Collect indicator data and give feedback from the perspective of ecological environment improvement. According to the obtained data, it can be used to analyze the ecological environment improvement performance, analyze the ecological environment improvement operation status, and diagnose the cause of the failure, and it can also be used to monitor the cause of the failure. Ecological environment improvement and real-time risk alerts are important manifestations of ecological environment improvement management and systematic integration, providing detailed data information for the operation and maintenance of ecological environment improvement. There is a certain value for the development of reflection from the perspective of green economy. If the reflection from the perspective of green economy reaches a certain value, environmental sustainability will grow in doubling manner. The areas that exceed this value are all distributed in the eastern region, followed by the middle area, and the area with the least value is located in the western range. With the continuous development of the Chinese green economy, the large-scale domestic green economy has developed rapidly, and more environmental sustainability communication channel projects have emerged [3, 4]. A detailed analysis of the environmental sustainability communication channels is carried out to explore the problems and shortcomings of the green economy development process. In the process of analyzing the development and evolution of green economy in traditional environmental sustainability communication channels, we usually mainly analyze the development and evolution of green economy in environmental sustainability communication channels. The current requirements of environmental sustainability communication channels require that environmental sustainability communication channel enterprises can solve a one-stop service system, provide strong support for life, and allow the entire environmental sustainability communication channel to obtain the highest economic benefits as the overall goal of sustainable communication channel enterprise work [5–7]. For the areas with frequent green economy business records in the early stage, it shows that the local communication technology level and communication business capabilities are relatively good, and the green economy is based on Internet technology, and the analysis of the development and evolution of the green economy in the environmental sustainability communication channel occupies an important position. A good green economic development and evolution analysis system can speed up the flow of environmental sustainability communication channels, reduce costs, and ensure the normal operation of services. In order to effectively improve the analysis accuracy of green economy development and evolution in the process of environmental sustainability communication channels, an evaluation algorithm is used to analyze the real-time evolution of goals in green economy development. Meanwhile, it will also bring more long-term benefits to various regions in the country [8–10]. By constructing a model, it evaluates the influencing factors between the development influencing factors and environmental sustainability of each regional economy. Therefore, it can be concluded that the accuracy of the sustainability of the green economy can be rapidly improved, and it can also promote the effective use of the green economy in various regions in China. By comparing the specific practices of other green economic development, an in-depth analysis of their commonalities and characteristics is conducted, to explore suitable paths for China's green economic development, and to provide solutions and theoretical basis for Chinese green economic development.

The development of green economy has gradually become an important research direction for the communication channel of urban environmental sustainability. Through in-depth analysis of typical green economic development models in China and foreign countries, the commonality and characteristics of its development process are explored, and the development process of building a green economy is effectively summarized, to effectively sum up the regularity and innovation in the process of building a green economy. Under the condition of fully grasping the principles of green economy rule of law and environmental sustainability and related policy protection, find out a suitable green economy rule of law and environmental sustainability model. At the same time, it can also start from the perspectives of the government, the market, and the public, and according to the needs of the market, industry-driven and technological innovation can be used as a strong support for the green economy, the rule of law, and environmental sustainability. Finally, the results of example analysis show that the evaluation algorithm used in this paper can effectively obtain high-precision green economy development goals evolution analysis results and meet the needs of real-time evolution analysis of green economy development analysis.

## 2. The Connotation of the Communication Channel of the Rule of Law and Environmental Sustainability

The rule of law acts as the basic requirement and effective path to effectively realize the modernization of the national management system. Using the channels of sustainable communication of the rule of law and the environment, under the influence of the channels of sustainable communication of the rule of law and the environment, the rule of law thinking will become the mainstream ideology in the future society, and the rule of law model will gradually become the basic method for the management of state institutions, government management, and social management [11, 12]. At different historical moments in history, the focus of the construction of the rule of law is different, which will make the content of legal thinking and the way of the rule of law present different characteristics. At present, the main focus of the rule of law thinking is to adhere to the premise of legality, combined with the ideology of rules, focus on judgments under the premise of adherence to legality, grasp the awareness of the rule of law, pay attention to procedural justice, and put the so-called “rule of law thinking” as the grasp of power, auditing the concept of the rule of law, conduct detailed analysis, reform, coordination, and other dimensions of problems in accordance with laws and regulations, legal principles, legal spirit, and legal thinking process, and analyze, summarize, judge, reason, and fully understand the process of decision-making thinking and cognition activities, using the rule of law thinking as the basis of the rule of law consciousness and the concept of the rule of law to achieve the sublimation of the theory, which has a guiding role in the improvement and practice of its legal system. The laws and regulations related to the rule of law and environmental sustainability are mainly based on the behavior patterns that emerge from the rule of law thinking, and the communication channel of the rule of law and environmental sustainability is the concrete embodiment of its content and form. As an effective ideological basis for the implementation of the rule of law in the environment, the rule of law thinking plays a decisive role in the way of the rule of law. The way of the rule of law is also the external manifestation and concrete content of the rule of law thinking, and it also fully embodies the rule of law thinking. In the construction of the rule of law management environment, the communication channels of the rule of law and environmental sustainability, especially for government organizations and their personnel, can avoid abandoning profit-seeking judgments instead of legality judgments when dealing with problems and reduce the use of policy thinking instead of law, reduce the use of policy thinking instead of legal rule thinking, which is specially used for understanding, analyzing, and discussing the concepts and rules of the rule of law, and better apply it in handling practical problems.

There are roughly two types of performance evaluations, that is, the evaluation of profitability and the evaluation of legality. Profitability evaluation, also known as utilitarian evaluation, is the degree to which the government can satisfy the basic functions of the government among many public and interest groups, that is, the actual performance of government governance and government management [13]. Generally speaking, the government must provide the people with the most basic security, order, and quality of life and build a people-centered social development framework. Otherwise, you will not have the support and approval of the people. It is self-evident that legitimacy needs the support of profitability. But it is dangerous to overexaggerate the role of economic performance and profitability in a legitimate construction. Huntington thought it was legitimate, hardworking proposition. In his view, the effort to establish legitimacy based on performance creates what is known as the performance dilemma. “Because their legitimacy is based on the standard of political performance, authoritarian regimes will lose their legitimacy if they cannot have good political performance, and if they have good political performance, they will also lose their legitimacy.” With performance as the sole source of legitimacy, if the government has good performance, such as achieving economic growth and social stability, the public may be concerned about other issues such as fairness, justice, subjective well-being, and personal development. If social productivity is an instrumental measure for judging the level of social development, then fairness, justice, subjective well-being, and human development are the value measures for judging the healthy and harmonious development of society. These are difficult to resolve or provide for regimes where performance is the only source of legitimacy. In fact, the sources of legitimacy include performance, jurisprudence, ideology, and personal qualities. In some respects, it is clearly not enough alone. Of these, legal compliance of conduct or social relationships is the most important source of legitimacy. The focus of the Rule of Law and Environmental Sustainability communication channel is the analysis of legitimacy, that is, all controversial actions, claims, interests, and relationships surrounding legal and illegal thinking and judgment. In this sense, in the context of the rule of law, the use of the communication channels of the rule of law and environmental sustainability requires first of all adherence to the priority of legality judgment rather than profitability judgment. The evaluation criteria for profitability are clear and highly maneuverable, but they only involve the surface and immediate aspects of government management. Judgments of legitimacy cannot be made in a short period of time but can be applied in all situations deemed beneficial to society, solving the problem fundamentally. In a word, only by adhering to the priority of legality judgment can we truly avoid modifying the values of the corresponding parameters as stated in the law on paper. The method in reality: American researchers have shown that the foundation of the rule of law lies in the fact that the government can act on citizens with faithful legal rules. The rules and laws that are referred to are what citizens need to abide by and must perform in their daily process. At the same time, as citizens' rights and obligations, they need to be announced and notified in advance under the effective rules. The purpose of making rules of the rule of law is a general guideline for popular behavior. From the perspective of rule of law thinking, the ideology of rules is the fundamental idea; if there is a lack of awareness of rules, there will be no reference basis for the communication channels of the rule of law and environmental sustainability. The coordination between Chinese economic growth and the ecological environment has been greatly improved, but the rate of improvement in each region is still very low, and there are large spatial differences in different regions. Therefore, in the process of promoting high-quality economic development, it is necessary to pay more attention and concern to environmental protection. Through the construction of a comprehensive evaluation index system for the coordinated development of economic growth and ecological environment, based on analyzing existing research theories, scientific and reasonable data, and information conditions, the development level of the regional economy is evaluated from the four perspectives of economic development, organizational structure, economic growth, and degree of economic openness. At the same time, the urban ecological environment quality is controlled from four aspects: resource use, environmental sustainability, urban greening, and pollution. The economic growth rate and the ecological environment are complementary and can be measured using the reflection from the perspective of the green economy.

## 3. Advancing a Green Economy Perspective Requires the Use of the Rule of Law and Environmental Sustainability Communication Channels

Improving environmental sustainability as the goal of economic development requires continuous improvement of environmental sustainability, so that economic development can have lasting momentum, and the steady development of society can have a solid foundation. However, because environmental protection usually lags behind economic construction, in the process of economic and social development, the incongruity phenomenon of the problem of “one leg is long and the other is short” often occurs in social development. The development of green economy activities is accompanied by the economic background and living environment. It can not only control the general direction in the form of currency, but also use the living environment to limit, promote the implementation of green economy, and make efficient use of resources [14, 15]. The so-called green economy is a new form of green economic activity that combines the traditional economy with computer Internet factors and digital technology to achieve investment, financing, payment, and security services. However, it is different from the traditional economy. The business of the green economy is more convenient, common, and efficient. It has the characteristics of the green economy, and its purpose is to develop the economy and the environment together. Through the role of economic development and living environment in the green economy, it is often expressed as stimulating consumers to consume, converting consumption concepts, and promoting economic models. Among them, Ant Financial Services and JD Green Economy can show that green economy enterprises can provide consumers with healthy and fast loans for consumption, stimulate consumers' purchasing and consumption needs, change the economic model, and shift from production-oriented to consumption-oriented. Among them, consumers prefer environmentally friendly products, such as energy-saving home appliances, green homes, and new energy vehicles. This preference has promoted the development of green enterprises, reduced negative economy, and improved the coordination between the rapid development of the economy and the environment.

Insurance, bonds, and funds in the green economy are used to raise more social funds and strengthen the amount of funds that can be actually used. By using cloud computing, it is possible to quickly identify the main loan data, carefully evaluate the loan risk of enterprises, and make full use of the green economic resources in the economic system. Liquidity hierarchy: the problem is that green economy capital facilitates the flow to more efficient and environmentally friendly sectors. For the real economy, “Blood transfusion” perfuses “real economy”—at the same time, it helps improve environmental benefits and further realize a virtuous circle of economic development and environmental improvement [16, 17].

The mathematical model is established as follows:

(1) $$\begin{array}{c} S_{t+n}=B_{t+n}\left(a,b\right)+V\left(a+\Delta a,b+\Delta b\right)+N_{t+n}\left(a,b\right). \end{array}$$

*B*_*t*_(*a*, *b*) and *B*_*t*+*n*_(*a*, *b*) represent the background of the green economy at frames *t* and *t* + *n*; V (a,b) and *V*(*a*+Δ*a*, *b*+Δ*b*) represent the environment sustainability communication channels at frames *t*, *t* + 1; *N*_*t*_(*a*, *b*) and *N*_*t*+*n*_(*a*, *b*) are the external disturbances of the green economy in frames *t*, *t* + *n*.

The t-th frame is obtained using the real-time update algorithm of economic data.

(2) $$\begin{array}{c} \Delta S_{\left(t+n\right)/t}=S_{t+n}-S_{t}=\left[B_{t+n}\left(a,b\right)-B_{t}\left(a,b\right)\right]+\\ \left[V\left(a+\Delta a,b+\Delta b\right)-V\left(a,b\right)\right]+\left[N_{t+n}\left(a,b\right)-N_{t}\left(a,b\right)\right] \end{array}$$

In the formula, [*B*_*t*+*n*_(*a*, *b*) − *B*_*t*_(*a*, *b*)]+[*V*(*a*+Δ*a*, *b*+Δ*b*) − *V*(*a*, *b*)] is the factor of green economy development channel; [*N*_*t*+*n*_(*a*, *b*) − *N*_*t*_(*a*, *b*)] is the factor of external interference.

H (a,b) represents the binary difference green economy of the real-time economic data update algorithm as shown as follows:

(3) $$\begin{array}{c} H\left(a,b\right)=\left\{\begin{array}{cc} 1, & \Delta S\geq N,\\ 0, & \Delta S<N. \end{array}\right. \end{array}$$

Among them, N represents the threshold.

If H (a,b) = 1, it means that the target in the video is in a green economic development state; if H (a,b) = 0, it means that the target is in a stationary state [18, 19].

Let Q (a,b) show the binary difference green economy after background update difference processing. Then,

(4) $$\begin{array}{c} Q\left(a,b\right)=\left\{\begin{array}{cc} 0, & \Delta S_{t/\left(t-1\right)}\cap \Delta S_{\left(t+n\right)/t}\neq 1,\\ 1, & \Delta S_{t/\left(t-1\right)}\cap \Delta S_{\left(t+n\right)/t}=1. \end{array}\right. \end{array}$$

If Q (a,b) = 1, it means that the channel point is in the green economic development area; if Q (a,b) = 0, it means that the channel point is in the background green economic development area, which means that it requires the background real-time update operation. Replace the background area with the channel of the *S*_*t*_ frame to realize the correction of the background channel.

(5) $$\begin{array}{c} B\left(a,b\right)=\left\{\begin{array}{cc} B_{m}\left(a,b\right)=S_{t}, & Q\left(a,b\right)=0,\\ B_{n}\left(a,b\right), & \text{otherwise.} \end{array}\right. \end{array}$$

Describe the updated background green economy *B*_*M*_ as the weighted sum of B and *B*_*m*_, that is,

(6) $$\begin{array}{c} B_{M}\left(a,b\right)=\delta \times B\left(a,b\right)+\left(1-\delta \right)\times B_{m}\left(a,b\right). \end{array}$$

The economic data real-time update algorithm conducts real-time evolution analysis of the environmental sustainability communication channel and uses the evaluation algorithm to accurately analyze the goals in the development of the green economy. *Y*_*k*_ represents the vector of the environmental sustainability propagation channel at time H, *C*_*k*_ represents the system observation vector, and then the environmental sustainability propagation channel state and observer can be expressed by the following formula:

(7) $$\begin{array}{c} Y_{k+1}=A_{\left(k+1\right)/k}Y_{k}+w_{k},\\ C_{k}=H_{k}Y_{k}+v_{k}, \end{array}$$

*w*_*k*_ represents the random external disturbance vector; *H*_*k*_ is the observation matrix; *v*_*k*_ is the observation external disturbance vector.

The evaluation algorithm is used to estimate the green economy development goals, and the estimation benchmarks are as follows:

(8) $$\begin{array}{c} J\left[{\tilde{Y}}_{k}\right]=J\left[Y_{k}-{\tilde{Y}}_{k}\right]=E\left[{\tilde{Y}}_{k}{\tilde{Y}}_{k}^{T}\right]=\min, \end{array}$$

where ${\tilde{Y}}_{k}$ is the unbiased estimate of *Y*_*k*_.

The vector evolution analysis and covariance equation of the a priori estimated green economy development goals are, respectively,

(9) $$\begin{array}{c} {\tilde{Y}}_{k+1}^{\prime }=A_{k+1}{\tilde{Y}}_{k},\\ Q_{k+1}^{\prime }=A_{k+1}Q_{k}A_{k+1}^{T}+P_{k}. \end{array}$$

The calculation formula of the gain matrix of the evaluation algorithm is

(10) $$\begin{array}{c} H_{k}=Q_{k}^{\prime }K_{k}^{T}{\left(K_{k}P_{k}^{\prime }H_{k}^{T}+G_{k}\right)}^{-1}. \end{array}$$

The vector update equation and the covariance update equation for the estimated green economy development goals are, respectively,

(11) $$\begin{array}{c} {\tilde{Y}}_{k}={\tilde{Y}}_{k}^{\prime }+H_{k}\left(C_{k}-K_{k}{\tilde{Y}}_{k}^{\prime }\right),\\ Q_{k}=\left(I-H_{k}K_{k}\right)Q_{k}^{\prime }. \end{array}$$

In the formula, ${\tilde{Y}}_{k+1}^{\prime }$ is the a priori estimated green economy development goal; *P*_*k*+1_′ is the estimated error variance matrix; the best estimated error variance matrix is *P*_*k*+1_; the coefficient matrix used for the best estimate is *K*_*k*_; ${\tilde{Y}}_{k+1}$ is the best estimate of the green economy development goal. As one of the three engines of economic development, green economy is closely related to the level of regional environmental management. The development of green economy can realize the economic adjustment of enterprises and enhance the coordination between economic growth and ecological environment by acting on the economic scale, economic efficiency, and economic structure of enterprises. First, in terms of economic scale adjustment, it can attract a large number of private capital and social capital into the green economy market, expand corporate financing channels, and increase corporate cash holdings. Alleviate the problem of insufficient green economy for enterprises, especially technology-based environmental protection enterprises. According to the research results, we can see the relationship between the growth of emerging economies and environmental sustainability. With the continuous increase of GDP per capita in various regions, the degree of environmental sustainability also experienced a first decrease, then an increase, and finally a downward trend [20, 21]. The economic analysis model constructed in each region conducts in-depth analysis on the evaluation of relevant economic development factors and evaluates the influencing factors between the development factors of each regional economy and environmental sustainability. The accuracy of the sustainability of the green economy can be rapidly improved and the efficient use of economic resources can also be promoted. Under the environment of green economy, while adjusting the economic structure of various regions quickly, it can provide an auxiliary role for environmental protection.

As a product of the rapid development of Internet technology, green economy has been proven in various fields as a new driving force for economic growth. He Bin invented a set of limit threshold models, which is aimed at the reflection of the per capita green economy perspective of each region in China and the impact of the state-owned economy on the improvement of the ecological environment. The key to the sustainable growth of the proposed economic development is to analyze the breakthrough in the economic structure and analyze it from the perspective of energy, which is actually the current situation provided by the current environment. Facts have proved that Chinese economic growth is inseparable from the two major causes of pollutant generation and environment in various regions of the country, especially for the huge Chinese market. Through two levels of analysis, the first level is that the economic resources of various regions in China are disparate, and the development of each region also has a large gap. The problems in the management of pollutant generation in various regions in China also need to take into account the growth of the economy.

## 4. Analysis of Example and Result

Based on the green and effective combination of economic development principles and models, this paper explores the potential laws of green economic development. Local governments, enterprises, and social groups are the key stakeholders in the communication channel of environmental sustainability, and their main goals and decisions will directly promote the development of green economy.  Figure 1 shows the decision-making process in the development of green economy through the construction of environmental sustainability communication channels [22].

Guided by the principles of green economy rule of law and environmental sustainability, the green economy development model can be illustrated in Figure 2.

This model can be roughly divided into three links, which are green economy and environmental sustainability composed of government-led, market adjustment, and public participation. The three links do not exist independently of each other but are linked and restricted. The function of the rule of law thinking and the rule of law model to the green economic development model and the relationship between the rule of law thinking show that the use of the rule of law and environmental sustainability communication channels has a crucial role in promoting the rapid development of the green economy. However, from the perspective of social life, due to their limited capabilities and different living environments, there are also differences in their ideals and beliefs, which will lead to a nonuniform green economy perspective, usually a state of diversification and dispersion. Under the premise of adhering to the concept of the rule of law, realize the understanding of various problems in the development of environmental sustainability, while using the principle of the rule of law to comprehensively evaluate and reason about environmental sustainability. It not only needs to be led and guided by relevant government departments, but also needs to be based on the degree of participation of social organizations. Act in accordance with the laws and regulations, and at the same time, according to the actual situation, adjust measures to local conditions and circumstances. Respond in a timely manner to policy adjustments for people-oriented environmental sustainability. Combined with this model, it is explained from the perspective of integrity and complexity, and the normative role of the communication channels of the rule of law and environmental sustainability is demonstrated by the analysis from the perspective of green economy.

The innovation of science and technology, as the driving force for the sustainable development of the digital economy, can form a virtuous circle between economic growth and environmentally sustainable development. Technological innovation is the key to a green economy. Through in-depth theoretical research and analysis, it can be seen that investment in science and technology can make economic growth form a scale effect and can promote productivity and sustainable economic development. Driven by the green economy, technological innovation can be applied and transformed to achieve higher economic growth. When formulating low-carbon emission reduction policies, it is necessary to effectively consider the basic economic development and social conditions, energy availability, and green related policies of each country, actively encourage countries to actively explore pollutant discharge and renewable energy quotas suitable for their own regions, and guide the whole society to save energy and improve energy efficiency to reduce environmental pollution. In the traditional economic and ecological environment analysis process, ecological environmental protection and real-time risk alerts are also effective data collection and analysis processes for ecological environmental protection. Collect indicator data from ecological environment protection and give feedback. According to the obtained data, it is used to analyze the performance of ecological environment protection, analyze the operation state of ecological environment protection, and diagnose the cause of failure and can also be used to monitor the cause of failure. Green economy promotes the upgrading of industrial structure by optimizing the allocation of credit funds, promoting technological innovation of enterprises, and enhancing consumer demand of residents. This in turn affects the interaction between the economic system and the environmental system. Specifically, for the manufacturing industry, which is the main body of the development of the real economy, the green economy arises from the development needs of the real economy. Network platforms and digital technologies are used to provide the manufacturing industry with better green economy services and improve the market structure of the green economy. Further support the green transformation of the economy. Ecological environment detection and real-time risk monitoring are of great significance for ecological environment-related resource distribution, flow planning service level, and safety monitoring.

## 5. Conclusion

Green economic development analysis has been widely used in green economic development. In order to further improve the accuracy of green economic development analysis of environmental sustainability communication channels, this paper proposes an environmental sustainability communication channel in terms of evaluation algorithms to help realize the analysis method of green economy development. The method collects economic data information for the objectives of the environmental sustainability communication channel process, fully considers the diversity of the environmental sustainability communication channel process, and analyzes the real-time evolution of the upgraded environmental sustainability communication channel. Combined with the evaluation algorithm to analyze the green economy development in the environmental sustainability communication channel, the experimental research shows that the method in this paper can accurately and quickly analyze the green economy development of the environmental sustainability communication channel process, which is relatively better than other evolution analysis methods, which can be used as a powerful tool for subsequent analysis of environmental sustainability communication channels.

## Figures and Tables

**Figure 1:** The main decision-making interaction of environmental sustainability communication channels for building green economy development.

**Figure 2:** Green economy development model.

## Data Availability

The data used to support the findings of this study are available from the corresponding author upon request.
